The article "Research on the Application of Blockchain in Smart Healthcare: Constructing a Hierarchical Framework" was retracted in 2023. Reasons: unreliable results or conclusions; concerns about the data; concerns about the peer review; concerns about the citations.

# Research on the Application of Blockchain in Smart Healthcare: Constructing a Hierarchical Framework

**DOI:** 10.1155/2021/6698122

**Published:** 2021-01-12

**Authors:** Xiaomin Du, Beibei Chen, Ming Ma, Yanjiao Zhang

**Affiliations:** ^1^Department of Economic Management, Yingkou Institute of Technology, Yingkou 115014, China; ^2^School of Economics and Management, Dalian University of Technology, Dalian 116024, China; ^3^Graduate School of Business, Changwon National University, Changwon 51140, Republic of Korea

## Abstract

This study aims to explore the application of blockchain technology in smart healthcare, establish a hierarchical theoretical framework of smart healthcare, reveal the impact of blockchain on smart healthcare, and finally, construct a development application system of smart healthcare under the blockchain based on stakeholder theory. However, such a hierarchical theoretical framework should consider not only the necessary attributes and the interrelationship among various aspects and attributes but also the role of multiple stakeholders. Therefore, the paper uses fuzzy set theory to filter unnecessary attributes, proposes a decision-making and experimental evaluation laboratory (DEMATEL) to manage the complex interrelationships between various aspects and attributes, and uses Interpretive Structure Modeling (ISM) to divide the hierarchy and construct a hierarchical theoretical framework. The results show that (1) the top-level design, the medical record management, and the doctor management are the root causes of system. (2) The specific application of blockchain in the field of smart healthcare is mainly carried out around the intelligent contract, which relies on the medical record management and is constrained by the system, and optimization of application is the key to system upgrading. (3) The internal and external regulation, the medical insurance, and the environmental governance play a guaranteed role for the development of the system and effectively safeguard the interests of stakeholders. (4) The application system of smart healthcare under the blockchain needs to be built based on three layers: the transaction layer, information layer, and stakeholder layer. The theoretical hierarchical framework is intended to guide smart healthcare towards blockchain applications, and stakeholders are suggested to participate in the development application systems.

## 1. Introduction

The rise of new technologies, such as Internet of Things and big data, has promoted the development and innovation of healthcare around the world and improved the construction of the smart healthcare system. Smart healthcare is a medical system with medical cloud data as the core, which combines electronic medical record, electronic health archive, and medical Internet of Things by using Internet of Things, data transmission, and exchange technologies to build medical and health services and optimal management. At present, the smart healthcare industry has made rapid progress, but there are still problems of information security and system security. As the key technology of the fourth industrial revolution [1], blockchain has the characteristics of decentralization, anonymity, tamper proof, and auditability [2]. The combination of blockchain and smart healthcare can alleviate the pain points of traditional smart healthcare in information sharing, data security, and privacy maintenance, optimize the user-centered smart healthcare systems, and establish a multiparty medical alliance chain involving government, enterprises, and individuals to promote the industrial upgrading of smart healthcare.

At present, blockchain has attracted the attention of the whole industry. Current research findings include basic blockchain bottom techniques [3, 4], blockchain key management [5], long-term verification analysis of blockchain signatures [6], and so on. But, the research on the application of blockchain in the smart healthcare field is not mature enough. Most of the existing studies are about the combination of blockchain and existing information technology to create a new data platform or data system, such as the construction of an electronic medical system based on blockchain [7, 8] and the building of a data privacy protection platform based on blockchain [9]. There are also some studies to explore the role of blockchain in the sustainable supply chain of smart healthcare from the perspective of supply chain, such as blockchain monitoring of counterfeit and substandard drugs [10, 11], blockchain monitoring of the operating environment of medical products [12], and integration and upgrading of blockchain to a supply chain system [13]. Although the abovementioned literature has made a deep research on the application of blockchain in the smart healthcare field, the development system of smart healthcare under the blockchain is not clear and still lacks the systematic research. Furthermore, the application of blockchain in the smart healthcare industry is hard to be explained clearly on an aspect because it will cooperate with all the subjects in the value chain of smart healthcare in the process of application and need multisubjects to coordinate and influence each other. However, from the perspective of stakeholders, exploring a multisubject coordinated development system is still rare. Finally, the existing application of blockchain in the field of smart healthcare mostly stays at the level of private chain and lacks of exploration at the level of alliance chain. Because the leading companies control the information, the information is not transparent enough in private blockchain and its application is limited [14]. Although, compared with the private chain, the public chain has a greater improvement in the credibility of information. However, the public chain needs to include many participants, and it is difficult to ensure the privacy and security of participants. In addition, it is “completely decentralized,” which hinders the design of the system. In contrast, the alliance blockchain has the characteristic of “partial decentralization,” and it is more conducive to the application of blockchain in the field of smart healthcare by adding limited main body in the application process to reduce the cost decrease risks and increase the trust degree.

Based on this, in order to develop the development and application system of the blockchain smart healthcare system based on alliance chain, the following research is carried out in this paper. Firstly, in order to totally study the impact of blockchain on smart healthcare, this study determines the composition of the stakeholders in the smart healthcare industry and their trading relationships from the perspective of stakeholders and combines the blockchain technology with it. Through exploration and collation, a set of 22 standards is proposed from ten aspects. Secondly, in order to clarify the importance of each attribute and sort out the dependence between attributes, it is necessary to consider the mutual restriction and influence of each attribute and, finally, make multiattribute decision. In the process, this study comprehensively uses fuzzy set theory, decision-making trial and evaluation laboratory (DEMATEL), and interpretive structural modeling (ISM) to evaluate the causality between attributes and discuss the interrelationships between various levels, revealing the influence path of blockchain on smart healthcare development. Finally, based on the abovementioned analysis and stakeholder theory, this study constructs a blockchain smart healthcare application system based on alliance chain from three levels: the transaction layer, information layer, and stakeholder layer.

The following scientific conclusions can be drawn in this paper. First of all, the improvement of blockchain to the smart healthcare system is mainly reflected in ten aspects, namely, top-level design, doctor management, medical records management, treatment optimization, community building, cost savings, internal and external regulation, medical insurance, and environmental governance. Secondly, the study found that these ten aspects have different importance. First, the top-level design, the medical records management, and the doctor management are the root causes of the system construction. Second, the specific application of blockchain in the field of smart healthcare is mainly around the intelligent contract, relying on the medical records management, constrained by the system, and optimizing the application is the key to upgrade the system. Third, regulation, medical insurance, and environmental governance play a protective role in the development of the system and effectively safeguard the interests of stakeholders. The internal and external regulation effectiveness is a decisive factor in the health of the system, and the implementation of health insurance and environmental governance needs to be promoted at the first three levels. Finally, the intelligent medical application system under the blockchain needs to be constructed based on three layers: the transaction layer, information layer, and stakeholder layer. The theoretical framework and application system in our research can not only provide the academia with cutting-edge theoretical references for the development of blockchain smart healthcare but also provide practical guidance for the smart healthcare industry on how to use blockchain technology.

## 2. Literature Review

Smart healthcare realizes the interaction between patients and medical staff, medical institutions, and medical devices by building a health archives regional medical information platform and using the most advanced Internet of Things technology, so that the medical industry gradually achieves information. Sharing medical data is an important step to make the medical system more intelligent and improve the quality of medical service [15]. However, the sharing of patient data among institutions is not yet fully realized [16], and the blockchain is a great way to solve this problem right now. Blockchain is distributed data systems involving multiple independent nodes [17], which is an emerging technology for decentralized and transactional data sharing among large networks of untrusted participants. It features decentralization, timestamps, collective maintenance, programmability, and tamper-proofing [18]. Blockchain has relatively few applications in medical treatment, and the existing research mainly focuses on combining blockchain with a certain information technology to build a single application platform, such as using blockchain technology to build a medical transaction sheet verification system; using etheric blockchain to build a medical information sharing platform MedRec which combines blockchain with big data [19]; and using blockchain technology and the OPAL/Enigma encryption platform to create a secure environment for medical information storage and analysis [20]. However, the application of blockchain technology in the whole intelligent medical industry lacks systematic research.

Based on this, the study will build a customer-centered blockchain smart healthcare application system based on stakeholder theory to explore its development path. After sorting out and analyzing all the stakeholders of the system, we get the application system based on ten aspects including 22 criteria.

### 2.1. Internal and External Regulation

Internal supervision mainly refers to the real-time supervision of drugs, equipment, and supply chain by medical institutions. External regulation includes three criteria: medical supply chain regulation, medical whole process regulation, and medical waste treatment process regulation, and the executive body is the regulatory body. The application chain is a system that involves the transfer of products or services from suppliers to customers, which is composed of people, organizations, activities, information, and resources. Its purpose is to ensure the quality of sensitive commodities throughout the shipment. Supply chain management is very important in the industry of transporting materials and goods. Also, drug supply chain management is particularly important for tracking the source of materials used for manufacturing, the process of manufacturing, and the distribution of finished products [21]. Centralized supply chain management systems expose supply chains to corruption, fraud, and tampering [22]. Effective supply chain management is particularly important in the medical field, where a compromised supply chain directly affects patient safety and health outcomes. One potential solution to improve the security, integrity, data sources, and functionality of a healthy supply chain is the blockchain technology [13]. In the supply chain, blockchain technology transactions are secure and transparent and can be permanently monitored and recorded, greatly reducing not only the time required but also the possibility of human error [23]. In addition, through the implementation of blockchain, the security of medical supplies and equipment can be improved. Blockchain technology can be achieved by saving unique device identifiers for each medical device and by tracking and publishing firmware updates using smart contracts. Blockchain-based medical device tracking can also use invariance to prevent device loss, theft, and malicious tampering [21].

### 2.2. Medical Record Management

Medical record management includes electronic medical record. Electronic medical record provides a convenient health record storage service that facilitates online electronic access to traditional paper medical records [24], which is highly sensitive information that needs to be shared among peers, to keep up-to-date patient history [25]. Current electronic medical record cannot ensure the security, privacy, and availability of sensitive data, and the patients' diagnosis and treatment data are still in a decentralized state in different medical institution databases [24, 25]. As a result, patients may lose control of available healthcare data, while medical institutions generally maintain primary management. Using blockchain technology to share electronic medical record is customer centered, and patients have the control of their electronic medical record. The decentralized, self-trusted, and tamper-resistant nature of the blockchain ensures the secure storage and delivery of medical data and greatly reduces the turnaround time for sharing and overall costs [26]. Also, because patients can participate in their own health records, they will focus more on their own healthcare [27].

### 2.3. Treatment Optimization

Treatment optimization includes two criteria: telemedicine and targeted therapy. The number of medical patients has increased dramatically in many countries, making it increasingly difficult for patients to obtain direct help from doctors or nursing staff [28]. Telemedicine technology is seen as a way to achieve equitable and cost-effective medical care [29]. The development and popularization of Internet of Things equipment and other remote patient monitoring systems have led to security risks in the transmission and recording of data transactions. Based on the characteristics of blockchain tamper-proof, anonymous, and transparency, the intelligent contract of the blockchain can be used to promote the security analysis and management of medical sensors [30]. For example, in Medical Chain, a smart contract has been launched through which patients can let doctors remotely review medical cases and provide suggestions or second opinions [23]. In addition, the data can be safely transmitted through blockchain asymmetric cryptographic encryption [17], and the drug research and development institutions classify the data after user authorization, so as to conduct drug-targeted research and development.

### 2.4. Doctor Management

The doctor management includes three criteria: identification, personnel screening, and customer selection. Blockchain technology allows for large-scale interoperability among healthcare providers, patients, and agents for information exchange, patient tracking, identity assurance, and authentication [31]. Besides, blockchain can be used to record doctors' treatment, so as to avoid medical disputes, thus facilitating medical institutions to select excellent doctors and patients to choose the right doctors. For instance, Medico Health is a blockchain-based project that allows completely anonymous and secure client communication with the world's leading physicians. Information on the validity of physician certificates and licenses is updated in an immutable decentralized database, and patient data are only stored and accessed anonymously by an appointed physician at a specified time [23].

### 2.5. Medical Insurance

The blockchain can provide a high degree of reliability for users due to its Practical Byzantine Fault Tolerance and multinode comaintenance nature [2]. AXA, France's leading insurance group, has started offering parameterized flight delay insurance based on its Ethereum platform called fizzyTM, which uses smart contracts connected to the global air traffic database to safely initiate compensation once flight delays are detected, thus avoiding the need for additional paperwork. A similar plan could be implemented for health insurance, eliminating the need to verify medical records and greatly simplifying the process [27]. The application of blockchain technology in medical insurance can reduce the complexity and cost of medical insurance [32], protect the interests of patients, and reduce the uncollected funds of hospitals and the management cost of insurance companies.

### 2.6. Cost Saving

Cost saving includes two criteria: the cost saving of doctor-patient communication and the cost saving of drug research and development. Credit Suisse's survey conducted in 2016 proved that hospitals, the pharmaceutical industry, and insurance companies could save money by implementing blockchain technology [27]. One of the main benefits of blockchain systems and electronic medical records is better access to medical records for both doctors and patients, improving nursing efficiency, and quality [33, 34]. Sharing a ledger among entities such as pharmacies and insurance companies can be extremely convenient for patient costs and medication management. Particularly in the context of chronic disease management, providing pharmacies with accurate updated data on prescriptions will improve logistics [26]. Multisite clinical trials at drug development facilities can reduce trial costs, while data management systems based on blockchain intelligent contract technology can reduce the cost of managing multisite clinical trials [35].

### 2.7. Top-Level Design

The top-level design includes three criteria: an industry standard, reward and punishment system, and credit rating system. The industry alliance organization formulates the industry standard uniformly, through the intelligent contract automation execution, and regulates the behavior of each node. The incentive mechanism is one of the core values of blockchain, which gives virtual currency rewards to those nodes that obey rules and punishes those nodes that do not. The incentive mechanism is an important part to make the application system develop benignly [36]. The industry alliance organization carries on the real-time regulation to this incentive mechanism, and gives the extra punishment to the main body which does not obey the rules. In addition, industry consortia can use blockchain technology to construct a credit rating system, urge the behavior of each subject, and reduce the cost of rating [37].

### 2.8. Community Structure

Community structure includes three criteria: health management, family sickbed and graded diagnosis, and treatment. Community is a support group of comforting the sick [38]. A private blockchain based on the Ethereum protocol creates a community healthcare system. Intelligent devices in users' homes can communicate with sensors, collect and upload residents' health data via the Internet of Things [28], and call smart contracts to record all events on the blockchain. The intelligent contract system sends notifications to patients and community doctors to support real-time patient monitoring and medical interventions, while maintaining a safety record of information about the people who initiated these activities [30].

### 2.9. Environmental Governance

Blockchain and its intelligent contract features have the potential to solve interoperability problems in the medical field, such as effective interaction between users and medical applications [39]. Blockchain technology can also be used to monitor waste and emissions in various steps of the supply chain [23]. In the process of medical waste treatment, the staff of each link can safely deliver the medical waste data to various organizations and equipment to improve the overall efficiency of the medical waste treatment process. The explicit explanation of each criterion is listed in Table 1.

## 3. Method

The fuzzy method can capture the fuzziness and complexity associated with the data. DEMATEL helps to deal with the complex relationships among selected standards. ISM can study the causal relationship among multiple criteria. Therefore, in order to obtain valuable results, the research combines the fuzzy set theory, DEMATEL, and ISM method. It explores from 10 factors to account for the internal correlation of the influencing factor system deeply, including external regulation (A1), medical record management (A2), treatment optimization (A3), doctor management (A4), medical insurance (A5), internal regulation (A6), cost saving (A7), top-level design (A8), community structure (A9), and environmental management (A10). Then, it uses the mixed DEMATEL means to standardize the mixed matrix and uses the matrix calculation to calculate a mixed integrated impact factor matrix. After that, we get the key factors of blockchain affecting smart healthcare by calculating its centrality and casuality.

### 3.1. Fuzzy DEMATEL

Fuzzy DEMATEL is a method that combines fuzzy mathematics and DEMATEL. The triangle fuzzy number (TFN) can transform our language preferences into a form that can be calculated. The DEMATEL technique is a practical and effective algorithm for influencing factor identification. In the traditional DEMATEL method, accurate numerical values are usually used to represent the intricate relationship between factors, which sometimes cannot fully reflect the real situation of the problem. In order to make up for the defects of the tradition DEMATEL method, the concept of TFN is introduced in the paper, and the fuzzy-mathematical method is proposed. This method increases the reliability of the evaluation results and becomes a more useful reference basis for managers to make decisions.

**Step 1 .**

In view of the research question, we construct the system influence factor system and set to F1, F2,…, F*n*.

**Step 2 .**

Expert scoring is used to determine the relationship between two factors and is expressed as a matrix. We design an expert evaluation semantic scale and divide the degree of influence among factors into 5 levels. See Table 2 for the specific degree of influence.

**Step 3 .**

By using the converting fuzzy data into the Cripps Scores (CFCS) method, the triangle fuzzy matrix and the direct influence matrix among the elements are obtained. The specific operation process of the CFCS method is as follows:

First, standardization of triangular fuzzy numbers:

(1) $$\begin{array}{c} xa_{1_{ij}}^{k}=\frac{a_{1_{ij}}^{k}-\min a_{1_{ij}}^{k}}{\Delta_{\min}^{\max}},\\ xa_{2_{ij}}^{k}=\frac{a_{2_{ij}}^{k}-\min a_{1_{ij}}^{k}}{\Delta_{\min}^{\max}},\\ xa_{3_{ij}}^{k}=\frac{a_{3_{ij}}^{k}-\min a_{1_{ij}}^{k}}{\Delta_{\min}^{\max}}. \end{array}$$

Second, we standardize the right-hand side and the left-hand side:

(2) $$\begin{array}{c} xls_{ij}^{k}=\frac{xa_{2_{ij}}^{k}}{\left(1+xa_{2_{ij}}^{k}-xa_{1_{ij}}^{k}\right)},\\ xrs_{ij}^{k}=\frac{xa_{3_{ij}}^{k}}{1+xa_{3_{ij}}^{k}-xa_{2_{ij}}^{k}}. \end{array}$$

Third, we calculate the clear value of each expert's score after it is blurred:

(3) $$\begin{array}{c} x_{ij}^{k}=\frac{\left[xls_{ij}^{k}\left(1-xls_{ij}^{k}\right)+xrs_{ij}^{k}xrs_{ij}^{k}\right]}{\left[1-xls_{ij}^{k}+xrs_{ij}^{k}\right]},\\ z_{ij}^{k}=\min a_{1_{ij}}^{k}+x_{ij}^{k}\times \Delta_{\min}^{\max}. \end{array}$$

Fourth, we calculate the average clarity value:

(4) $$\begin{array}{c} z_{ij}^{k}=\frac{\left(z_{ij}^{1}+z_{ij}^{2}+\cdots +z_{ij}^{k}\right)}{n}. \end{array}$$

**Step 4 .**

We standardize the direct influence matrix *Z*:

(5) $$\begin{array}{c} \lambda =\frac{1}{\max_{1\leq i\leq n}\sum_{j=1}^{n}z_{ij}},\;G=\lambda Z. \end{array}$$

**Step 5 .**

On the basis of *T*=*G*+*G*^2^+⋯*G*^*n*^ or *T*=*G*(*E* − *G*)^−1^, *E* is the constant matrix, and the composite impact matrix *T* is taken.

**Step 6 .**

The degree of influence and being influenced are the values obtained by adding each row and each column of the composite impact matrix. The calculation formulas are

(6) $$\begin{array}{c} D_{i}=\sum_{j=1}^{n}t_{ij}, \end{array}$$

(7) $$\begin{array}{c} R_{i}=\sum_{i=1}^{n}t_{ij}. \end{array}$$

The sum of the influence degree and affected degree is called centrality, representing the role of elements in the system. The difference between the influence degree and the affected degree is called causality. The calculation formulas are

(8) $$\begin{array}{c} m_{i}=D_{i}+R_{i},\;\left(i=1,2,\ldots ,n\right), \end{array}$$

(9) $$\begin{array}{c} n_{i}=D_{i}-R_{i}, \end{array}$$

### 3.2. ISM

ISM can transform fuzzy ideas and viewpoints into intuitionistic models with good structural relations. Then, the direct influence matrix is calculated to obtain a comprehensive influence matrix. An all-inclusive influence matrix *t* reflects only the mutual influence relationship and degree between different factors, without considering the influence of factors on itself. Hence, calculating the overall impact relationship of system factors is critical and needful. The calculation process is as follows:

(10) $$\begin{array}{c} H=T+E=h_{ij};\\ \lambda =\alpha +\beta , \end{array}$$

where *α* and *β* are the mean and standard deviation of all elements in the synthetic impact matrix *T*, respectively.

We determine the reachable matrix between the factors.

(11) $$\begin{array}{c} M={\left[m_{ij}\right]}_{n*n},\;\left(i=1,2,\ldots ,n;j=1,2,\ldots ,n\right), \end{array}$$

(12) $$\begin{array}{c} m_{ij}=\left\{\begin{array}{c} 1,\;h\geq \lambda ,\\ 0,\;h\leq \lambda . \end{array}\right. \end{array}$$

If there is a relationship between element *i* and element *j*, then the value is 1; otherwise, it is 0.

Through layered processing, the reachable set *L*(*f*_*i*_), the antecedent set *P*(*f*_*i*_), and the common set,

(13) $$\begin{array}{c} C\left(f_{i}\right)=L\left(f_{i}\right)\cap P\left(f_{i}\right), \end{array}$$

are obtained.

At last, the reachable set and the general set determine the ISM model.

## 4. Results

On the basis of literature review and analysis, this paper summarizes 10 factors influencing blockchain-based intelligent medical treatment. From August to October 2020, we selected, in a serious manner, seven people who have worked in the healthcare industry for more than 10 years as our interviewees. We conducted a field survey on them and obtained their mutual influence on these 10 influencing factors through face-to-face interviews. We revised and summarized their answers to obtain the fuzzy direct impact matrix, then used the CFCS method to process the original data, and determined the direct impact matrix of the influential factors of blockchain technology in intelligent medical treatment, as shown in Table 3.

To standardize the direct impact matrix of smart healthcare blockchain technology, we obtain the standardized direct influence matrix. Then, we obtain the comprehensive impact matrix based on the *T*=*G*(*E* − *G*) − 1 and the calculation of MATLAB, as shown in Table 4.

Equations (6)–(9) can be used to obtain the influence degree, affected degree, centrality, and causality, as shown in Table 5.

We make a causal diagram, as shown in Figure 1. Figure 1 is a visual representation of the data in Table 5. From Figure 1, we can clearly see the centrality and causality of the factors.

The ten risk factors are separated into a cause set and a result set based on the degree of the cause, and it is shown in Table 6. There are seven reasons, including A8 top-level design, A2 medical record management, A4 doctor management, A3 treatment optimization, A5 community structure, A7 cost saving, and A6 internal regulation. Among them, A8 top-level design, A2 medical record management, and A4 doctor management are the main motivations. The influence degree of A2, A4, and A8 is 2.3122, 2.4441, and 2.4071, respectively, which are the three most influential factors, manifesting that these three factors have the greatest impact on other factors. This is because top-level design, medical record management, and doctor management are the roots of the impact of blockchain on smart healthcare. There are three result elements, including A1, A5, and A10, which have little impact on smart healthcare but are more susceptible to other factors. So, in practical management, these factors should be taken into account and placed under appropriate control to improve management effectiveness. For centrality, these factors follow the order of top-level design (A8), doctor management (A4), medical record management (A2), cost saving (A7), external regulation (A1), treatment optimization (A3), community structure (A9), internal regulation (A6), medical insurance (A5), and environmental management (A10).

The reachable matrix obtained from formula (12) is shown in Table 6.

Through the reachable matrix and formula (13), the first-order decomposition structure is calculated, as shown in Table 7.

As shown in the table above, the accessible set and public set intersect at factors A5 and A10, so elements A5 and A10 become first-order impact factors. We delete the rows and columns mapped by the influencing factors A5 and A10 in the matrix *M* to obtain a higher level decomposition matrix. By analogy, the factors at all levels are obtained. The subsets *N*_*q*_(*q*=1,2,3,4) of each layer are finally obtained through several levels of division: first-level node *N*_1_={5,10}; second-level node *N*_2_={1,6}; third-level node *N*_3_={3,9,7}; and fourth-level node *N*_4_={4,2,8}. Based on the abovementioned analysis, the paper can establish the ISM as shown in Figure 2.

Based on the ISM analysis, top-level design (A8), medical record management (A2), and doctor management (A4) are the first elements that blockchain influences smart healthcare, and the key is to determine how to monitor and control these factors in a timely manner.

To sum up, the factors influencing the application of blockchain in the sustainable development of smart healthcare are complicated. However, the method of influence, mechanism of influence, and degree of action differ depending on the factors, so a system integration framework for the development of sustainable intelligent medicine under the blockchain was prepared, and a scientific application framework was sought.

## 5. Discussions

This study tries to explore the intelligent medical development system based on blockchain technology. Blockchain technology has not been fully applied in the domain of smart healthcare and lacks a comprehensive hierarchical model. This study proposed a series of standards for the smart healthcare system and built a hierarchical model.

All the transactions in the system are executed on the intelligent contract, which is a kind of computer protocol designed to spread, verify, or execute the contract in the way of information, and it improves the transaction efficiency by its automatic execution, thus reducing transaction costs [40]. First of all, top-level design, medical record management, and doctor management are at the first level of the ISM model, with the highest centrality, which is also the root of the impact of blockchain on smart healthcare. The top-level design, including the development of industry standards, rewards and punishments system, and the rating system, is located at the top layer of the framework and plays an overall role. Its main aim is to ensure the authenticity of the source data and to prevent companies from being induced to engage in joint fraud [41], at the same time, to prevent the disadvantages of a lack of applications, infrastructure, and services that go with the blockchain [42], strengthen the policy subsidies in this area, and use blockchain technology for more comprehensive and reliable, convenient, and efficient quality certification and credit evaluation. Therefore, the top-level design plays a guiding role in the entire system. To develop and improve the blockchain smart medical system, we must first improve the top-level design. Medical record management runs through the entire blockchain smart medical system. An electronic medical record is vital and highly sensitive personal information in healthcare that needs to be shared frequently among peers [26]. In this study, a blockchain-based electronic medical record sharing system is proposed, which provides security for medical data and private information and overcomes the shortcomings of electronic medical records in traditional intelligent medical services. Customers have access to and copy of their own electronic medical records, which can be easily licensed to other medical institutions or third-party platforms [43]. Note that the client only has read-only permissions, and the doctor has to upload and modify permissions under the premise of client authorization. The management of doctors further deepens the client-centered idea of the system. Blockchain technology can realize the interoperability of the identity assurance and verification of patients and medical staff [31]. We use blockchain to build a verification platform to verify the identity and certificates of doctors on a regular basis, so as to ensure the safety of patients and high-quality medical care. At the same time, the blockchain is used to collect and update the doctors' diagnosis results and correct rates, which is convenient for hospitals to select excellent doctors and also conducive to customers' accurate medical treatment.

Treatment optimization, community construction, and cost saving belong to the second level, which are the concrete application of blockchain in the system. Treatment optimization includes targeted therapy and telemedicine. Based on the abovementioned information, customers have the right to manage their own data [43]; drug research and development institutions can obtain the required customer data after customer authorization and payment of fees and can conduct targeted drug research and development after collation and analysis. Based on the integration of blockchain and the Internet of Things technology, smart devices are linked to sensors; the telemedicine system can help patients and medical institutions to proactively respond to medical conditions through near real-time monitoring and treatment, improve the quality of medical treatment, and reduce the cost of medical treatment [44]. Community construction includes health management, family sickbed, and grading diagnosis and treatment. In this community medical system, sensors communicate with smart devices, collect and upload health data of residents through Internet of Things technology and wearable smart devices [28], and call smart contracts to write records of all transactions on the blockchain. An intelligent contract system sends notifications to patients and community physicians to support real-time monitoring of patient and medical interventions, while also keeping a security record of who initiated these activities [30]. Based on this, the community doctor first carries on the first-level diagnosis and treatment to the resident and decides whether patients need to go to the hospital for further treatment according to the situation, saving the cost of residents' medical treatment. In addition, smart contracts can be used to build community health projects based on residents' health data, which is conducive to residents' health maintenance. The cost saving includes the cost saving of doctor-patient communication and the cost saving of drug research and development. Sharing medical data through blockchain helps patients with medication and cost management and is an important step in making the medical system more intelligent and improving the quality of medical care [15, 26]. The data-sharing system in the system consists of trusted peers—medical institutions, patients, and other third parties. Multiple medical institutions cooperate to execute consensus agreements and maintain a distributed ledger, and patients can access and manage their data through applications on any node that stores their information. The key management processes and access control policies are coded as a chain code to protect security and patient privacy [26]. The implementation of multisite clinical trials for drug research and development institutions can reduce the cost of trials, while the data management system based on blockchain smart contract technology can reduce the management costs of multisite clinical trials [35].

Internal and external regulation belongs to the third level, and its effectiveness is the crucial factor for the healthy development of the system. Data on the supply chain of medicines and medical devices are publicly available because the safety of medical supplies and medicines in the supply chain directly affects the health and safety of users, and everyone has the right to know [45]. The traceability, tamper-resistance, and transparency of blockchain make it a key monitoring technology for the entire movement of drugs and medical products [46]. Blockchain technology ensures that the general ledger chain of transactions is immutable and tracks every step of the supply chain at a single drug level [47], eliminating the production and trafficking of counterfeit medicines and illicit products. Besides, the whole medical process and medical waste disposal process will also be uploaded to the public chain through the Internet of Things technology, and their behaviors will be constrained by intelligent contracts. The supervision department will conduct real-time supervision and form a joint supervision force.

Health insurance and environmental governance belong to the fourth level, and their implementation needs the first three levels of common promotion. They are also the last level of application of blockchain to the smart medical system. Health insurance includes two components: resource control and improving risk management ability. In this system, patients' treatment data and insurance company's payment are uploaded to the blockchain in real time, reducing fraud in medical insurance claims [48]. Medical institutions upload and store the consumption data of patients into the blockchain, and multiple nodes work together to ensure the accuracy of the uploaded data. The insurance company can know the sum of the expenses through the authorization of patients, but cannot know the details of the expenditures, protecting the interests of patients while protecting their privacy [49], while also reducing the hospital's unpaid bills. Environmental governance refers mainly to the treatment of medical waste, and blockchain enables effective interaction between users and medical applications [39]. Hospitals and medical waste treatment institutions cooperate inside and outside and use technologies such as blockchain and Internet of Things to strictly control the medical waste treatment process. The person in charge of each link will upload medical waste production data, handover records, and treatment data (desensitization) to the public blockchain to ensure medical waste data can be traced back to the source and, at the same time, attach upload person, upload time, and upload data to ensure the credibility of the data.

This study further develops the blockchain smart healthcare application system based on alliance chain combined with the conclusion of ISM model analysis, so as to understand the hierarchical framework of this study totally (Figure 3). The system is divided into an transaction layer, information layer, and stakeholder layer. Considering the characteristics of small radiation range of private chain, easy control, and poor privacy of public chain, this paper chooses the alliance chain with high operability and reliability [50]. From the abovementioned analysis, top-level design is the key and foundation, and its construction cannot be separated from the government's formulation and promotion of related policies. Based on stakeholder theory, this study proposes that the application of blockchain technology is deployed and controlled by 11 participating nodes in the federated layer of the alliance chain; these nodes are customers, medical institutions, doctors, communities, drug research and development institutions, institutional review committees, suppliers, regulators, insurance companies, medical waste treatment institutions, and industry consortia, the 11 participating nodes form a stakeholder layer. The transaction relationship between different nodes is analyzed, and the transaction information between the two parties is determined to constitute the information layer. With the blockchain as the carrier, the stakeholder layer deals with the information layer on the smart contract to form the transaction layer. Blockchain is a large database of transaction information in the system. The feasibility and security of each transaction are guaranteed by the multinode joint maintenance and traceability. The information in the federation chain is divided into public information and private information according to the degree of authorization of the nodes, and the blockchain uses the public-key cryptography technology to encrypt the information [51], so the security coefficient of private information is higher.

## 6. Conclusions

Current research in the area of smart healthcare focuses on single information technologies such as the Internet of Things in healthcare [39], but currently, patient data cannot be safely shared between institutions, and privacy protection has become a bottleneck in today's intelligent health industry [52]. Of course, there are some studies that combine blockchain with smart medical care, but most of them focus on the application of a certain characteristic of blockchain in the field of smart medical care [30, 53, 54], and the research subjects are mostly patients and medical institutions. Few studies consider multiagent cooperative development and lack the application system of smart healthcare development under the blockchain. Compared with the previous research, this study explores the multilevel development path of blockchain in the field of smart healthcare based on stakeholder perspective, and the final application system of blockchain TIS is more explicit and total. The comprehensive application of fuzzy methods, DEMATEL methods, and ISM methods can filter out the necessary attributes and manage the complex interrelationships between various aspects and attributes.

However, the study still has a few limitations. Firstly, although the criteria constructed in this paper are selected through a broad literature review, they still cannot contain all possible attributes. Secondly, the expert group is composed of smart medical management professionals. However, the committee should include experts in other relevant fields, especially blockchain technology, to expand its scope and application. Therefore, a more comprehensive discussion with experts in the future to explore a more effective solution of block chain for intelligent medicine, as an extension of the existing hierarchical framework, is the focus of future work. Thirdly, though the study uses fuzzy set theory to eliminate the subjective bias of experts, it is not deep enough. Moreover, other analysis tools can also be used in this study for a more comprehensive exploration. Finally, the data of this paper are mainly from China. Future research can explore a more perfect and diversified blockchain intelligent medical governance framework based on different cultural and technical backgrounds.

## Figures and Tables

**Figure 1:** DEMATEL causal diagram.

**Figure 2:** ISM structure model.

**Figure 3:** TIS application system based on alliance chain.

**Table 1:** Proposed attributes.

Aspects	Criteria	Explanation
External regulation (A1)	Medical supply chain regulation	The regulation department supervises the drug and equipment supply chain through the blockchain
	Medical process regulation	Regulators monitor medical processes through the blockchain
	Regulation of clinical waste treatment process	The medical waste disposal process is monitored by the regulatory authority through the blockchain

Medical record management (A2)	Electronic medical record	Using blockchain technology to share electronic medical records; customers have absolute ownership

Treatment optimization (A3)	Targeted therapy	Using blockchain technology to share patient data; drug discovery agencies are licensed to target drugs
	Telemedicine	The use of blockchain and Internet of Things and other technologies for telemedicine

Doctor management (A4)	Identification	Using blockchain technology to build a verification platform, the doctor's identity, and certificate for periodic verification
	Personnel screening	Using blockchain to collect and update the diagnosis results and correct rate of doctors in real time and to screen the excellent doctors
	Customer choice	Using blockchain to store the doctor's identity information and treatment information; it is also helpful for customers to choose the right doctors

Medical insurance (A5)	Maintenance of interests	Insurance companies, customers, and medical
	Resource control	Institutions through the blockchain intelligent contract insurance transactions to protect the interests of customers
	Enhancing risk management capacity	Reduce the hospital's unpaid bills

Internal regulation (A6)	Regulation of drugs and medical equipment	Using the blockchain to set up a tracking system; medical institutions can monitor the flow of drugs and medical equipment in real time

Cost saving (A7)	Cost saving in doctor-patient communication	Using blockchain to share electronic medical records and saving communication cost
	Cost saving of drugs research and development	Data management system based on blockchain intelligent contract technology to reduce the management cost of multisite clinical trials

Top-level design (A8)	Industry standards	Industry associations establish industry standards
	Credit rating system	All nodes are rated by the industry consortia
	Reward and punishment system	The node that obeys a rule is given reward, and the node that does not obey a rule is given punishment

Community structure (A9)	Health management	Using blockchain to collect customer health data and create community health programs
	Family sickbed	Using blockchain and Internet of Things technologies for remote monitoring and treatment at home
	Hierarchical diagnosis and treatment	Community doctors perform primary care, analyzing the patient's physical condition and deciding whether to go to a hospital

Environmental management (A10)	Clinical waste treatment	Through blockchain and Internet of Things technology to upload medical waste treatment data and improve treatment efficiency

**Table 2:** Semantic translation.

Language variable	TFN
N (no effect)	(0, 0, 0.2)
VL (very low impact)	(0, 0.2, 0.4)
L (low impact)	(0.2, 0.4, 0.6)
H (high impact)	(0.4, 0.6, 0.8)
VH (very high impact)	(0.8, 1, 1)

**Table 3:** The direct influence matrix of blockchain technology on smart healthcare.

	A1	A2	A3	A4	A5	A6	A7	A8	A9	A10
A1	0	0.1690	0.0167	0.1690	0.6833	0.0167	0.0167	0.1690	0.0167	0.6833
A2	0.0167	0	0.4357	0.4929	0.4167	0.3595	0.4357	0.4167	0.5500	0.3214
A3	0.5690	0.4548	0	0.1310	0.4357	0.0548	0.4548	0.2833	0.3024	0.2071
A4	0.3024	0.1310	0.5690	0	0.3024	0.2262	0.5690	0.4167	0.5690	0.2071
A5	0.0167	0.0548	0.0167	0.0167	0	0.0167	0.0167	0.0738	0.0167	0.0167
A6	0.4738	0.1310	0.0738	0.2262	0.4929	0	0.0738	0.2452	0.2262	0.4357
A7	0.5500	0.2452	0.4167	0.0738	0.0167	0.1119	0	0.2643	0.0167	0.2262
A8	0.2452	0.4548	0.4357	0.4929	0.2452	0.4548	0.4167	0	0.4929	0.3024
A9	0.5690	0.1310	0.0167	0.1310	0.3976	0.6833	0.1690	0.1310	0	0.4357
A10	0.0167	0.0548	0.0167	0.0167	0.0167	0.0167	0.0167	0.0738	0.0167	0

**Table 4:** The comprehensive impact matrix of blockchain technology on smart healthcare.

	A1	A2	A3	A4	A5	A6	A7	A8	A9	A10
A1	0.0440	0.0861	0.0483	0.0835	0.2414	0.0433	0.0501	0.0902	0.0473	0.2369
A2	0.1878	0.1190	0.2390	0.2394	0.3037	0.2186	0.2497	0.2378	0.2523	0.2648
A3	0.2382	0.1022	0.0728	0.1019	0.2344	0.0727	0.1880	0.1486	0.0650	0.2028
A4	0.2678	0.2362	0.2773	0.1256	0.2958	0.1908	0.2886	0.2458	0.2599	0.2564
A5	0.0183	0.0254	0.0166	0.0163	0.0170	0.0162	0.0173	0.0311	0.0161	0.0205
A6	0.1986	0.1293	0.0865	0.1233	0.2405	0.0575	0.0892	0.1352	0.0681	0.2178
A7	0.2383	0.1037	0.1769	0.1123	0.1874	0.0905	0.0777	0.1453	0.0849	0.1789
A8	0.2480	0.2377	0.2435	0.2466	0.2783	0.2435	0.2495	0.1413	0.2428	0.2759
A9	0.2437	0.1068	0.0685	0.1043	0.2395	0.2386	0.1085	0.1132	0.0556	0.2412
A10	0.0183	0.0254	0.0166	0.0163	0.0216	0.0162	0.0173	0.0311	0.0161	0.0159

**Table 5:** Comprehensive impact matrix analysis.

Factor	Influence degree	Affected degree	Centrality	Causality
A1	0.9712	1.7031	2.6743	−0.7319
A2	2.3122	1.1718	3.4840	1.1404
A3	1.4265	1.2459	2.6724	0.1806
A4	2.4441	1.1696	3.6137	1.2745
A5	0.1948	2.0596	2.2544	−1.8648
A6	1.3461	1.1878	2.5339	0.1582
A7	1.3959	1.3358	2.7318	0.0601
A8	2.4071	1.3197	3.7268	1.0875
A9	1.5199	1.1081	2.6280	0.4118
A10	0.1948	1.9111	2.1059	−1.7163

**Table 6:** Reachable matrix.

*M*	A1	A2	A3	A4	A5	A6	A7	A8	A9	A10
A1	1	0	0	0	1	1	0	0	0	1
A2	0	1	1	1	1	1	0	1	1	1
A3	1	0	1	0	0	1	0	0	0	0
A4	1	1	1	1	1	0	0	1	1	1
A5	1	0	0	0	1	0	1	0	0	0
A6	1	0	0	0	1	1	1	0	0	0
A7	0	0	0	0	0	0	0	0	0	0
A8	1	1	1	1	1	0	1	1	1	1
A9	0	0	0	0	1	0	0	0	1	1
A10	0	0	0	0	0	0	0	0	0	1

**Table 7:** First-level decomposition structure.

*I*	*L*(*f*_*i*_)	*P*(*f*_*i*_)	*C*(*f*_*i*_)=*L*(*f*_*i*_)∩*P*(*f*_*i*_)
A1: external regulation	8, 9, 10	1, 3, 4, 5, 6, 8	8
A2: medical record management	1, 2, 3, 4, 5, 6, 9, 10	1, 2, 3	1, 2, 3
A3: treatment optimization	4, 8	1, 2, 3, 4	4
A4: doctor management	1, 2, 3, 4, 5, 6, 8, 9, 10	1, 2, 3	1, 2, 3
A5: medical insurance	9	1, 2, 3, 5, 7, 8, 9	9
A6: internal regulation	7, 9	1, 5, 7	7
A7: cost saving	6, 8	1, 2, 3, 6	6
A8: top-level design	1, 2, 3, 4, 5, 6, 7, 8, 9, 10	1, 2, 3	1, 2, 3
A9: community structure	5, 7, 8, 9, 10	1, 2, 3, 5	5
A10: environmental management	10	1, 2, 3, 5, 8	10

## Data Availability

Data used to support the findings of this study are available upon request.
